# Adrenal Schwannomas: Rare Tumor of the Retroperitoneum

**DOI:** 10.1155/2015/547287

**Published:** 2015-05-26

**Authors:** Emanuele Grasso, Michele Simone

**Affiliations:** Department of General Surgery, Santa Maria Clinic, Via De Ferrariis 22, 70124 Bari, Italy

## Abstract

Schwannoma is a benign neurogenic tumor originating from Schwann cells. These produce the myelin sheath that covers peripheral nerves that are often affected. This latter localization is extremely rare, and only a few case reports can be found in the medical literature. Studies have shown that approximately 0.5% to 5% of schwannomas are retroperitoneal, constituting 0.2% of adrenal incidental tumors. These usually present as incidental findings, nonsecreting adrenal masses in asymptomatic patients. Diagnosis of a schwannoma is based on detection of spindle cells with Antoni A and Antoni B regions in histological sections and positive staining for S-100 protein by immunohistochemical analysis. We report a case of an incidentally identified during an abdominal ultrasound examination with schwannoma localized in the left adrenal gland.

## 1. Introduction

Schwannoma is a benign neurogenic tumor originating from Schwann cells. These cells produce the myelin sheath that covers peripheral nerves often affected.

However, schwannoma arising from the adrenal gland is an extremely rare entity. Additionally, it may arise from the retroperitoneal space, spinal nerves, and less frequently the adrenal medulla [1, 2].

This latter localization is extremely rare, and only a few case reports can be found in the medical literature. Studies have shown that approximately 0.5% to 5% of schwannomas are retroperitoneal, constituting 0.2% of adrenal incidental tumors [3].

These usually present as incidental findings, nonsecreting adrenal masses in asymptomatic patients.

Most often malignant schwannomas are associated with neurofibromatosis types 1 and 2 [4]. Histologically, they are distinguished by the presence of areas with high and low cellularity, called Antoni A and Antoni B.

Diagnosis of a schwannoma is based on detection of spindle cells with Antoni A and Antoni B regions in histological sections and positive staining for S-100 protein by immunohistochemical analysis [5].

We report a case of an incidentally identified during an abdominal ultrasound examination with schwannoma localized in the left adrenal gland. A brief review of the corresponding literature is also presented.

## 2. Case Report

A 45-year-old man was referred to our institution with a retroperitoneal left adrenal mass that was incidentally found by ultrasound 3 mo earlier. His medical history revealed mild hypertension under medication and an operation of appendicectomy 37 y earlier. He had no remarkable family history. Physical examination of his abdomen revealed no palpable mass. The patient had no cutaneous lesions or palpable lymphadenopathy.

Routine blood tests of the patient were normal, and the 24 h urinary catecholamines, cortisol, and chromogranin values were within normal ranges.

Ultrasonography demonstrated a 12 cm in maximal diameter heterogeneous expansive mass near the left adrenal. A computed tomography (CT) scan of the abdomen confirmed the ultrasound finding and revealed a 14 cm diameter heterogeneous mass with both solid and cystic components arising in the right adrenal gland (Figure 1).

Taking into account the size of the tumor and after informed consent was received from the patient, the authors proceeded with surgical treatment.

The patient underwent a laparotomy resection of the lesion, as well as an en bloc excision of the left adrenal gland. Histological examination of the resected specimen revealed macroscopically globular mass with areas of necrotic colliquation, measuring 14 cm (Figure 2).

Microscopic examination showed that the lesion was composed of Antoni A areas, where short spindle cells with a long conical nucleus and scant cytoplasm aggregated and formed a spiral structure, and Antoni B areas, where inflammatory cells were scattered within a loose matrix.

In immunohistochemical analyses, the tumor did not stain for c-kit (CD117), CD34, or SMA but stained strongly for S-100 protein and CD68 (Figure 3; 4).

The patient, whose postoperative course was uneventful, was dismissed on the fifth postoperative day. Ultrasonic and CT checkups at 6, 12, and 18 months showed no signs of recurrence.

## 3. Discussion

The majority of the tumors originating in the adrenal medulla are pheochromocytoma, neuroblastoma, or ganglioneuroma. Schwannoma of the adrenal gland is rarely encountered, although it similarly originates from the cells of the neural crest.

The origin of the adrenal schwannoma is considered to be either of 2 myelinated nerve systems innervated to the adrenal medulla: one is the sympathetic nerve from the upper lumbar plexus and the other is the phrenic or vagus nerve [6].

Schwannomas constitute approximately 1% to 5% of all retroperitoneal tumors. Malignant degeneration of a schwannoma is infrequent; however, when it occurs, it acts as a high-grade sarcoma with a high probability of causing local dissemination and distant metastasis.

Generally, malignant forms are suggested histologically by increased mitosis, pleomorphism, and vessel infiltration. Malignant schwannomas are typically found in the extremities, and often they occur in association with Von Recklinghausen's disease [7]. Although schwannomas can occur at any age, they predominantly occur in females between the second and fifth decade of life. In the retroperitoneum, these tumors are most commonly found in individuals between 40 and 60 y of age, with a slight female predominance (male/female ratio 2 : 3) [7, 8].

Preoperative diagnosis of schwannoma of the adrenal gland is often incidental, because large, deeply situated tumors are usually present for long periods of time before patients complain of symptoms. The size of lesions at the time of diagnosis is frequently >4 cm in diameter. However, the size of the lesion and the depth of invasion are not associated with the possibility of malignancy [9]. Patients commonly present often misleading symptoms such as nonspecific and mild abdominal pain or simply abdominal distension, depending on the size and location of the lesion.

In cases of retroperitoneal schwannomas that appear to localize in the adrenal glands, the differential diagnosis, which may be made by magnetic resonance imaging (MRI), ultrasonography, and CT, includes tumors of the area, such as adenoma of the adrenal gland, pheochromocytoma, myelolipoma, metastatic lesion, neurofibroma, paraganglioma, lipoma, and malignant fibrous histiocytoma [7]. Preoperative diagnosis is difficult, however, because these imaging techniques are nonspecific for demonstration of pathognomonic features unique to this lesion. It is imperative in circumstances with adrenal lesions in which the clinician excludes the presence of a hormone-releasing tumor, especially pheochromocytoma [9].

In cases of retroperitoneal lesions, MRI is the imaging modality of choice, because it allows better demonstration of their origin, vascular architecture, and relation to surrounding structures. MRI typically demonstrates benign schwannomas as well-circumscribed homogeneous masses that enhance slightly after intravenous administration of contrast material. Moreover, MRI shows low signal intensity on T1-weighted images and high signal intensity on T2-weighted images. These findings, although nonspecific, are commonly exhibited by schwannomas and have been reported to be present in 57% of the cases [10].

However, imaging modalities cannot provide a definitive diagnosis. Surgical resection of the lesion is necessary to make the diagnosis, differentiate it from other soft tissue neoplasms, palliate symptoms, and eliminate the possibility of malignancy. Biopsy is not recommended as a diagnostic tool, because hemorrhage, infection, and seeding of tumor cells are known risks of this modality, as are the lethal consequences if a pheochromocytoma exists [7].

Conventionally, schwannoma are divided into 2 distinct subtypes: hypercellular “Antoni A” type and hypocellular “Antoni B” type. Spindle cells are arranged in fascicles in areas of high cellularity with little stromal matrix in the Antoni A type. Nuclear-free zones called “Verocay bodies” can also be found in between the regions of nuclear palisading. Tumor cells are less densely found, forming loose meshwork often accompanied by microcysts or myxoid changes in Antoni B type, and are considered to be a degenerated form of the Antoni A type [6].

Both subtypes can be found as a mixture in adrenal schwannoma; 3 of 11 reported cases demonstrated both subtypes in a tumor. The differential diagnosis made using immunostaining should exclude gastrointestinal stromal tumor (GIST) or leiomyoma. Schwannoma positively stains for S-100. By contrast, GIST is positive for c-kit, and leiomyoma is positive for smooth muscle actin.

As evident from the medical literature, schwannomas that arise from the adrenal medulla are very rare entities. Often, schwannomas from the retroperitoneum, especially in the juxta-adrenal space, can be misdiagnosed when they mimic adrenal lesions [9]. In Poland, among 1111 adrenal incidentalomas, only 2 (0.18%) patients appeared to have schwannomas [3]. Fewer than 20 adrenal schwannomas are reported in the literature and 2 cases were identified during autopsy [11].

The ages of the patients ranged from 11 to 89 y, and no sex predilection was observed. The size of the lesions that are reported varies between 0.6 cm and 14 cm. All of the lesions are characterized by benign features [2–4, 9].

The common surgical approach that was followed was laparotomy and complete excision of the mass and the adrenal gland, with controversy existing over the necessity of negative margins, especially when adjacent tissues were in close proximity. In one case, partial adrenalectomy took place. In less than half of the cases, the patients underwent laparoscopic excision.

## 4. Conclusion

Retroperitoneal schwannomas are rare tumors that are difficult to diagnose. Preoperative workup is nondiagnostic and can only postulate a nonsecreting adrenal mass.

Schwannoma of the adrenal glands is a very rare entity, which in the vast majority of cases possesses benign behavior. This lesion is found predominately incidentally, and the clinician must have a high index of suspicion to recognize it when special features are demonstrated in imaging modalities, especially MRI. Histological and immunohistochemistry analyses provide the definitive diagnosis.

A nonsecreting adrenal mass >4 cm in diameter should be removed surgically with an added benefit of a definitive diagnosis.

The common surgical approach that was followed was laparotomy and complete excision of the mass and the adrenal gland while in the partial adrenalectomy the patients underwent laparoscopic excision.

## Figures and Tables

**Figure 1:** Computed tomography showing a 14 cm, well-circumscribed, enhanced round tumor with solid and cystic components arising in the right adrenal gland.

**Figure 2:** Photograph showing the gross appearance of the resected encapsulated tumor.

**Figure 3:** 4 Microscopic view showing benign schwannoma cells, along with alternating Antoni A and Antoni B patterns with fibrinoid degeneration, thrombosis, and hyalinization (H&E, magnification_100).
